RETRACTED

# Evaluation of the green economic value added index in the game of enterprise capital providers

**DOI:** 10.1016/j.heliyon.2023.e23890

**Published:** 2023-12-18

**Authors:** Wunhong Su, Quansheng Zhang, Yunxia Ling, Wong Ming Wong

**Affiliations:** a School of Accounting, Hangzhou Dianzi University, Hangzhou, Zhejiang, China; b International College, Krirk University, Thailand

**Keywords:** Green economic value added, Capital providers, Game theory

## Abstract

This study explores the performance evaluation of steel enterprises, emphasizing the importance of green environmental performance. Based on the review of the current situation of green investment research, economic added value evaluation system, and game analysis of enterprise capital providers, this study discusses the comprehensive evaluation of games among enterprise capital providers from the perspective of green economic added value. It constructs a game model of capital providers from the perspective of green investment. This model is based on the probability of creditors making green bond investments and shareholders pledging equity, deriving game results, and using economic added value returns to measure enterprise performance. The main data in this study are from the CSMAR database, a corporate governance project, and the relevant environmental protection data from Nangang's annual report. The results show that the green economic added value return rate is higher than the traditional economic added value return rate, indicating that environmental investments do not reduce the operational performance of enterprises. The game of capital providers leans towards equity investment and does not enhance enterprise performance at the expense of the environment. The green economic added value index only reflects past operational performance, based on which enterprises can design reasonable performance evaluation mechanisms, encouraging capital providers to favor environmental investments. This study has important theoretical and practical significance, guiding enterprises' strategic choices during green transformation.

## 1 Introduction

With the increasing frequency of environmental problems, people are paying more and more attention to corporate social responsibility, environmental protection, and green development. The output of Chinese iron and steel enterprises is at the forefront of the world, and studying Chinese iron and steel enterprises can provide a good reference. By discussing the performance evaluation of iron and steel enterprises, this study constructs a game model of capital providers from the perspective of green investment, hoping to explore ways for enterprises to improve green performance while operating profits, protect the earth's environment, and achieve sustainable development of human beings.

RETRACTED

Negative externalities of environmental issues and self-interested behaviors of enterprises lead to environmental pollution (Smith, 2020). Green environmental protection and innovation investments are low due to these negative externalities and uncertainties (Johnson et al., 2021). Nevertheless, the prior study has found a long-term equilibrium relationship between renewable energy consumption and economic growth (Lee, 2022). China's environmental policy has shifted from a pollution prevention perspective to an ecological civilization one, integrating economic measures like carbon trading markets and environmental taxes (Chen & Wang, 2023). The environmental hearing system and the “Public Participation in Environmental Protection Act” foster public participation in environmental governance (Liu et al., 2023). The pollution prevention campaign's evolution from the “Thirteenth Five-Year Plan” to the “Fourteenth Five-Year Plan” indicates deeper, more complex, and broader issues requiring amplified efforts (National Development and Reform Commission, 2024). The “National Plan for the Protection of Important Ecosystems and Major Projects” provides environmental development stage guidelines [1]. These initiatives positively influence the interplay between enterprise capital providers from the perspective of Green Economic Value Added (GEVA) (Zhang, 2026).

China has incorporated resource and environmental loss into GDP calculations, reflecting the environmental cost of economic development [2]. While sustainable development has become a global trend, green investments increase enterprise costs and necessitate improved resource utilization, reduced pollutant emissions, and production equipment upgrades [3]. However, replacing fossil resources with renewable ones presents challenges due to the instability of renewable energy, which necessitates the complementary use of thermal power generation [4]. China faces substantial pressure in ecological and environmental protection, striving to achieve peak carbon emissions by 2030 and the Beautiful China goal by 2035 [5]. Enterprises’ separation of ownership and control leads to agency problems, and conflicts of interest between shareholders and creditors form a game [6]. Different performance evaluation indicators impact the interplay among capital providers [7]. EVA is a new performance evaluation metric reflecting comprehensive enterprise financial management development [8]. These measures actively promote the interplay between enterprise capital providers from the GEVA perspective [9].

RETRACTED

This study explores the interplay among enterprise capital providers during the green transition, focusing on the game between creditors and shareholders in green investment decisions [10]. Using Nanjing Iron and Steel Co., Ltd. as a case study, this study examines how creditors and shareholders influence GEVA through game analysis [11]. Theoretically, this study introduces GEVA into the game analysis to compensate for the traditional EVA's neglect of the environmental impacts of enterprise activities [12], thereby better realizing the enterprise's sustainable development strategy [13]. The interplay between creditors and shareholders determines whether the enterprise makes environmental investments [14]. Green investments are not only the need for market development but also a necessary means to enhance an enterprise's sustained competitiveness and achieve socially sustainable development [15]. Therefore, the game choices of enterprise capital providers help enterprises make wiser strategic choices in their green transition [16].

This study employs game analysis, comparative analysis, and case study methods to explore the behavior of enterprise capital providers in green investment decisions. First, the Nash equilibrium probabilities of creditors and shareholders in green investments are forecasted through game analysis [17]. Then, leveraging comparative analysis introduces the concept of GEVA [12], emphasizing the importance of environmental cost in enterprise performance evaluation [18]. Finally, using Nanjing Iron and Steel Co., Ltd. as an example [19], the probability of making green investments and the investment return rate are analyzed through game theory [20] and the GEVA model. This is compared with the traditional EVA [21], further verifying the necessity for enterprises to invest in green environmental protection projects [22].

Nash equilibrium is an important economic concept that refers to a situation in which each player chooses the optimal strategy given an opponent's strategy. In game theory, Nash equilibrium probability is often used to study strategy choice and market equilibrium. Comparative leverage analysis evaluates the risks and benefits of different companies by comparing their financial leverage. It can help investors compare the financial conditions of different companies to make more informed investment decisions. Using methods such as Nash equilibrium probability and comparative leverage analysis can help us better understand economic decisions and the functioning of markets.

Nash equilibrium probability can be used to study the strategic choice of an individual or firm in a complex market environment, while comparative leverage analysis can be used to evaluate a firm's financial condition and risk. These methods can not only help us understand the principles of microeconomics but can also be used to formulate macroeconomic policy. Using Nash equilibrium probability and comparative leverage analysis can help us better understand economic decisions and market operations and formulate more effective economic policies. Therefore, this paper uses Nash equilibrium probability and leverage comparative analysis to explore the behavior of corporate capital providers in green investment decisions.

RETRACTED

Starting from the green context of China's goals for peak carbon emissions and carbon neutrality [23], this study innovatively explores the financing strategies of enterprises during their green transition from the perspective of the interplay between shareholders and creditors [24]. Furthermore, it incorporates environmental costs into the EVA performance evaluation system [25]. Furthermore, this study establishes a GEVA evaluation model [26], an improvement over the traditional EVA, demonstrating that the return on GEVA surpasses that of traditional EVA [27]. Finally, it focuses on sustainable enterprise development [28] and advocates for green enterprise transition under the impetus of green government policies [1].

Compared with previous studies, while focusing on the game of enterprise capital providers, this study introduces the concept of GEVA, emphasizes the importance of environmental protection and sustainable development, and adopts the method of a comprehensive evaluation to conduct a comprehensive analysis. GEVA evaluates a company's financial performance, considering all capital costs. There are limitations and computational difficulties in practical application. Calculations require complex financial analysis and market data, and accounting processes affect the results. Ignoring non-financial factors makes a full assessment impossible. Note that different capital cost rates and discount rates apply to different companies and industries, are based on historical data, and do not reflect future changes and uncertainties. Green EVA is an evaluation tool and is not a substitute for other methods and tools. It is necessary to conduct comprehensive analysis and decision-making with other methods and tools and pay attention to the conditions and scope of use to avoid abuse and misuse. By exploring the performance evaluation of iron and steel enterprises, building a game model, and analyzing and discussing the game results, it is of great significance for enterprises to choose financing strategies for green environmental protection actions, assume social responsibilities, and provide theoretical and practical value for future research.

RETRACTED

This study discusses the behavior of corporate capital providers in green investment decisions, which is of great significance for enterprises in choosing financing strategies, taking green and environmental actions, and actively undertaking social responsibilities. It provides reference and inspiration for enterprises to make wiser strategic choices. This study adopts game analysis and other research methods to systematically explore the behavior of enterprise capital providers in green investment decision-making, which provides theoretical and practical value for future research, deepens the green investment theory, and provides important references for enterprises’ strategic decision-making.

This study unfolds over five sections, revolving around GEVA and the interplay among enterprise capital providers: the introduction outlines the research background, significance, methodology, and conclusions, concurrently introducing the concept of GEVA. First, the theoretical research section lays the foundation for the study based on four theories. Second, in the model establishment section, a capital provider model is constructed through the interplay of shareholders and creditors, with Nash equilibrium calculations used to determine game outcomes. Third, the case study section uses Nanjing Iron and Steel Co., Ltd. as an example to calculate the GEVA and analyze the impact of the interplay among capital providers. Finally, the conclusion and policy recommendation section summarizes the research results, proposes specific suggestions, and reflects upon the study.

## 2 Literature review

### 2.1 Current state of research

Corporate environmental investment involves allocating funds to environmental protection activities to maintain ecological balance and achieve sustainable economic and environmental development (Bansal & Roth, 2000). The emphasis enterprises place on green performance is influenced by industry differences, and green performance has become a new standard for evaluating an enterprise's operational condition (Schaltegger & Wagner, 2006). However, environmental investments can lead to short-term financial burdens, especially poor economic returns (Chen, Chang, & Lee, 2015). In addition, environmental tax systems and pollution fee systems may impact corporate environmental investments by increasing the cost of pollution, thus encouraging enterprises to participate in environmental governance (Pigou, 1920). Meanwhile, the relationship between corporations and the environment is seen as either a “win-win” or “alternatively mutual gain” [18]. The former emphasizes that environmental investments can enhance an enterprise's production efficiency and competitiveness, while the latter suggests that environmental investments could increase costs and affect competitiveness. CSR plays an important role in shaping corporate investment behavior and efficiency, and a high level of CSR participation can reduce investment inefficiency and thus improve investment efficiency [29].

RETRACTED

Since its introduction by Stern Stewart & Co. in 1982, the EVA model has been widely used to measure corporate performance [12]. EVA has gradually attracted the attention of scholars both domestically and internationally, with research covering its impact on stock prices, superiority over traditional financial indicators, and role in promoting corporate innovation capabilities (Biddle, Bowen, & Wallace, 1997; Kim, 2006). Some studies apply the economic value-added approach to real-life corporate data and demonstrate the value of companies through case studies [30]. At the same time, the emergence of GEVA has enhanced the assessment of environmental performance (Makri & Endaya, 2019).

The GEVA is crucial in considering corporate ecological benefits and comprehensive costs, particularly in high-energy consumption and high-pollution enterprises (Chen, Ong, & Hsu, 2010). In the long run, EVA can enhance corporate value and encourage autonomous innovation, and constructing a GEVA model requires considering environmental costs [12]; Makri & Endaya, 2019). Green innovation is influenced by natural, economic, and policy factors (Kammerer, 2009). It can promote regional economic growth and social welfare (Cainelli, Mazzanti, & Montresor, 2012), Corporate innovation can promote environmental performance [31], and government subsidies can stimulate enterprises to undertake green innovation (Lee, Park, Yoon, & Park, 2010). Environmental taxes and pollution fees promote green innovation (Lambert & Silva, 2012). They can optimize resource allocation, drive industrial upgrades, and reduce environmental pollution (Fullerton & Metcalf, 2001).

Game analysis is important in helping decision-makers make more informed and rational decisions and avoid potential risks and conflicts. In market competition, game analysis helps enterprises understand competitors' strategies and behaviors to better cope with market changes. One study analyzed the asymptotic stability of equilibrium and explored the mechanisms that influence the system's evolution to an ideal state by constructing a tripartite evolutionary game model of government, enterprise, and energy regulatory service centers [32]. The study found that government subsidies should be gradually weakened under appropriate penalties to achieve carbon reduction goals, and enterprises should be guided to innovate independently to achieve a green and low-carbon economy. Another study examined the strategic behavior of local government, capital, and people by constructing a tripartite evolutionary game model [33]. This study attempts to combine evolutionary game theory and scenario analysis methods to provide a new perspective for upgrading industrial structures and the green development of the regional economy and promote industrial structure upgrading and sustainable development.

RETRACTED

Research indicates that the interplay between shareholders and creditors can affect corporate decisions and the balance of interests (Myers, 1977). Measures such as judicial remedies and environmental regulations can modulate the outcomes of this interplay (Pargendler, 2016; Darnall, Henriques, & Sadorsky, 2010). Managers and significant shareholders influence corporate value through various means (Shleifer & Vishny, 1986). Establishing a system resulting from multiple negotiation rounds and protecting creditors’ interests is crucial to achieving equilibrium [14]. The phenomenon of controlling shareholders infringing on investor interests is widespread (La Porta, Lopez-de-Silanes, Shleifer, & Vishny, 2000), and green investment is the result of multi-party negotiation, where government subsidies and market mechanisms play a significant role (Brunnermeier & Cohen, 2003). Over time, companies issue green bonds, the proceeds of which are used to fund climate-friendly projects. These bonds are becoming more common, and investor response to issuance announcements has been positive, with issuers improving their environmental performance after issuance and companies credibly demonstrating their commitment to the environment for initial and third-party certified bonds [34].

To sum up, based on the perspective of GEVA, this study analyzes the game relationship between capital providers and enterprises from the perspective of GEVA by building a game model. It discusses the comprehensive evaluation of the game of enterprise capital providers from the perspective of GEVA, hoping to promote the sustainable development of the economy, environment, and society. It also provides some reference for the financing methods of heavy-polluting enterprises.

### 2.2 Theoretical foundations

The development of game theory provides a theoretical foundation for the dynamic interplay between corporate development and environmental protection (Neumann & Morgenstern, 1944). The contradiction between a corporation's pursuit of economic benefits and environmental protection determines whether it will make green investments (Ambec & Lanoie, 2008). Simultaneously, the game among stakeholders, such as shareholders and creditors, also influences corporate decisions (Admati & Pfleiderer, 1994). Environmental regulations, clean technology, and policy support can effectively enhance a corporation's environmental performance, though adherence to regulations often leaves room for improvement (Gray & Deily, 1996; Popp, 2006). Recent studies have constructed a multi-agent game model, revealing the trade-offs between environmental protection and economic benefits among governments, corporations, and the public (Keser & Gardner, 1999; Lopez, Sterner, & Afsah, 2000). The green transition is seen as the optimal strategy for enterprises, and GEVA is used to measure corporate performance (Bennett, James, & Klinkers, 1999). Through game theory, it is found that the carbon tax levied by the government is more effective in encouraging low-carbon manufacturing than government subsidies for low-carbon technologies [35]. The outcome of the game depends on whether both parties can reach a consensus, affecting the game's effectiveness (Brandenburger & Nalebuff, 1995).

RETRACTED

Environmental costs refer to the price of environmental damage caused during the production process, including the expenses of remedial measures and the overdraft of future environmental protection costs (Tietenberg, 1994). This also involves the optimal allocation of resources and considerations of economic and ecological rationality (Pearce, Markandya, & Barbier, 1989). Environmental value manifests in natural, positive, negative, and daily consumption values, among other aspects (Costanza et al., 1997). Internalizing environmental costs involves incorporating environmental protection costs into the price of goods, with the responsibility for remediation borne by those who damage the environment (Pearce, 1993; Fullerton & Metcalf, 2001).

The Triple Bottom Line theory underscores the balanced consideration of economic, social, and environmental benefits (Elkington, 1997). Economic benefits pursue cost savings and revenue growth, but this should not be at the expense of the environment (Freeman, Harrison, & Zyglidopoulos, 2018). Environmental benefits consider the impact of human behavior on environmental quality and work to prevent the tragedy of the commons, though it can be challenging to measure these benefits accurately (Hardin, 1968; Costanza et al., 1997). Social benefits measure the impact of economic activities on social welfare, including aspects such as people's health and quality of life (Dasgupta, 2001; Chiu & Yang, 2017). Green economic interventions can positively impact these benefits, but innovation-driven development often lags [18]; Kemp, 2010). Therefore, enterprises should aim to balance economic, social, and environmental benefits through green equipment and technological innovation, thereby addressing the negative externalities and tragedy of the commons associated with the environment (Stavins, 2003; Acemoglu, Aghion, Bursztyn, & Hemous, 2012).

RETRACTED

EVA is the profit obtained after subtracting the equity and debt capital cost from net income after tax. An important indicator accurately reflects an enterprise's operating performance [12]. EVA emphasizes innovation and investment in sustainable development, encourages improved asset management and profitability, and has a ‘memory’ function guiding enterprises to create value continuously (Kim, 2006; O'Byrne, 1996). It serves as the basis for performance evaluation and financial management, providing a foundation for the incentive compensation of operators (Tursoy & Faisal, 2018; Cordeiro & Sarkis, 2008).

Stakeholder theory stresses that a corporation, functioning as a coalition of stakeholders, must balance the rights and interests of shareholders, creditors, suppliers, consumers, the government, and environmental standards (Freeman, 1984; Donaldson & Preston, 1995). Within the extant principal-agent relationship, the transparency of information and the cost of controlling agents can help minimize agency costs (Eisenhardt, 1989; [6]. Building on traditional EVA, GEVA integrates environmental factors to holistically measure the residual value produced by corporate operations (Hart & Milstein, 2003). It emphasizes sustainable development and a green ecosystem, contemplates ecological benefits, and incorporates environmental opportunity costs when evaluating corporate performance [36]. This approach propels green development in corporations, promoting a balanced progression of the economy and environment [18].

Corporate Social Responsibility (CSR) theory underscores that while striving for shareholder value, corporations must also accept responsibility for their impacts on society and the environment (Carroll, 1991). Corporations should stimulate industry competitiveness and technological innovation while meeting civic obligations (McWilliams, Siegel, & Wright, 2006; Porter & Kramer, 2006). Corporations voluntarily disclose social responsibility reports, elucidating environmental expenditures and measures, thereby promoting environmental investment and adherence to social responsibility (Dienes, Sassen, & Fischer, 2016; Clarkson, 1995). Moreover, CSR can foster green innovation, and attention from the media and government regulation can further propel environmental investment (Flammer, 2013; Peloza, 2009). Although green investment may escalate short-term costs, it is advantageous for long-term corporate growth. This necessitates policy support and external supervision, coordination of relations with all stakeholders, and the attainment of dual objectives of economic profit and environmental preservation [14]; Bansal & Roth, 2000).

RETRACTED

## 3 The impact of capital providers’ game on GEVA and model establishment

### 3.1 The game between Shareholder equity pledging and creditor green bond investment

Green bond investments can help reduce corporate pollutant emissions and improve environmental quality. Although their returns may be delayed and uncertain, good environmental performance can enhance corporate reputation and rebuild market confidence [34]. However, equity pledging might lead major shareholders to focus on short-term returns too much, which is detrimental to long-term development (Chen, Harford, & Lin, 2018). When societal norms emphasize corporate social responsibility, environmental performance can provide greater reputational protection for corporations (Barnett, 2007; Du, Bhattacharya, & Sen, 2010). Green investment is a crucial means to reduce pollution emissions and a strategy for reputation management. However, equity pledging may signal poor corporate performance, potentially reducing investment in the corporation (Billett, King, & Mauer, 2007).

Creditors and shareholders hope the enterprise can make profits and prevent bankruptcy; therefore, their interests are largely aligned. To ensure the maximum benefits of invested capital, shareholders and creditors must supervise corporate operators [6]. While protecting their interests and reducing transaction risks, they focus on the enterprise's risk resistance and debt repayment capabilities (Myers, 2001).

Creditors seek financial security and prefer stable returns of principal and interest. At the same time, shareholders pursue excess returns and prefer high-risk, high-return investments, leading to a difference in their risk-bearing capacities [6]. Shareholders' equity pledging might hint at financial issues, triggering a tendency in corporations towards green investment and exhibiting myopic behavior (Chen, Harford, & Lin, 2018). Creditors’ green bond investments, which may be delayed and uncertain, aim to improve their reputation [34]. This creates a game model that uses EVA and GEVA to measure corporate performance, revealing the impact of financing methods on performance [12,36].

The green assessment of Nansteel Shares helps to fulfill social responsibility. A corporate value evaluation model based on GEVA considers environmental investment. When GEVA exceeds zero, shareholders still have residual income after deducting all costs. Conversely, if GEVA is less than zero, it suggests that operating income cannot cover costs. Therefore, GEVA and corporate shareholder value change in the same direction [12,36].

RETRACTED

This study defines the following parameters: NOPATt denotes the Net Operating Profit After Tax for period t. GEVAt represents the Green Economic Value Added for period t. gEVAt signifies the adjusted Green Economic Value Added for period t. $\Delta I_{t}$ denotes the total new investment for period t. The corporation's value equals the initial total capital plus the present value of the expected GEVA.

The equation is expressed as:

(1) $$Corporate\;value=I_{0}+\sum_{t=z}^{\infty }\frac{GEVA_{t}}{{\left(1+WACC\right)}^{t}}$$

Calculated from equations (3)–(1), we obtain:

$$\text{Corporate}\;\text{Value}=I_{0}+\sum_{t=1}^{\infty }\frac{\left(NOPAT_{t}-I_{t-1}*WACC\right)+gEVA_{t}}{{\left(1+WACC\right)}^{t}}$$

$$=\sum_{t=1}^{\infty }\frac{NOPAT_{t}}{{\left(1+WACC\right)}^{t}}+I_{0}-\sum_{t=1}^{\infty }\frac{I_{t-1}*WACC}{{\left(1+WACC\right)}^{t}}+\sum_{t=1}^{\infty }\frac{gEVA_{t}}{{\left(1+WACC\right)}^{t}}$$

$$=\sum_{t=1}^{\infty }\frac{NOPAT_{t}}{{\left(1+WACC\right)}^{t}}+I_{0}-\sum_{t=1}^{\infty }\frac{I_{t-1}}{{\left(1+WACC\right)}^{t-1}}+\sum_{t=1}^{\infty }\frac{I_{t-1}}{{\left(1+WACC\right)}^{t}}+\sum_{t=1}^{\infty }\frac{gEVA_{t}}{{\left(1+WACC\right)}^{t}}$$

$$=\sum_{t=1}^{\infty }\frac{NOPAT-\Delta I+gEVA_{t}}{{\left(1+WACC\right)}^{t}}$$

Financing corporate shareholders through equity pledging might convey adverse signals, potentially leading to short-term behaviors that can affect corporate reputation (Bharath, Sunder, & Sunder, 2008). Conversely, creditors enhance corporate reputation and recover their invested capital through green bond investments [34]. However, the uncertainty and costs associated with green investments must be considered (Horvathova, 2010). The game between shareholders and creditors is determined by changes in equity pledging and decisions related to green bond investments (Bolton & Freixas, 2000).

Assume the following.

(1) The total cost for creditors to invest in green bonds is C (Baker, Greenwood, & Wurgler, 2003);
(2) The good reputation brought to the enterprise by creditors' green bond investments leads to a profit of P for the enterprise [34];
(3) The revenue obtained by shareholders through equity pledging is A [6];
(4) The loss caused by the adverse signals conveyed by shareholders' equity pledging to the market is K (Bharath et al., 2008);
(5) The revenue brought by shareholders' long-term innovative investments instead of pledging equity for short-term objectives is F (Bolton & Freixas, 2000);
(6) The probability that creditors' green bond investments will increase compared to last year is α, and the probability that it will not increase is 1-α (Khan, Serafeim, & Yoon, 2016);
(7) The probability that shareholders will increase the amount of equity pledged compared to last year is β, and the probability of not increasing the equity pledge is 1-β (Hansmann & Kraakman, 2001);

The game matrix between shareholders and creditors is shown in Table 1 as follows.

RETRACTED

**Table 1:** Creditor and shareholder game matrix.

	Shareholder Increases Equity Pledge (Shareholder) β	Shareholder Does Not Increase Equity Pledge (Shareholder)（1-β）
Creditor Increases Green Bond Investment (Creditor) α	-C + P,A-K	-C, F + K
Creditor Does Not Increase Green Bond Investment (1-α)	-P, A + K	0,0

Table by authors. Due to the large number of forms, we put the subsequent forms in the appendix.

The expected return for the creditor is as follows:

(2) $$E_{g}\left(\alpha ,\beta \right)=\alpha \left[\beta \left(-C+P\right)+\left(1-\beta \right)\left(-C\right)\right]+\left(1-\alpha \right)\left[\beta \left(-P\right)+\left(1-\beta \right)0\right]$$

Therefore, the expected return for the creditor when the investment in green bonds increases (a = 1) and when the investment in green bonds does not increase (a = 0) are respectively calculated by equation (2) as follows:

$$E_{g}\left(1,\beta \right)=\beta \left(-C+P\right)+\left(1-\beta \right)\left(-C\right)=\beta P-C$$

=(0,β)=βA+(1−β)0=−βP

$$E_{g}=\left(1,\beta \right)=E_{g}\left(0,\beta \right)\;\text{Let}$$

βP−C=−βP

$$\beta =\frac{C}{2P}$$

The formula for calculating the expected return of shareholders is as follows:

(3) $$E_{e}=\left(\alpha ,\beta \right)=\beta [\alpha \left(A-K\right)+\left(1-\alpha \right)\left(A+K\right)+\left(1-\beta \right)[\alpha \left(F+K\right)]$$

The expected return of shareholders, calculated by substituting into equation (3), is as follows:

$$E_{e}=\left(\alpha ,0\right)=\alpha F+\alpha K$$

$$E_{e}=\left(\alpha ，1\right)=-2\alpha K+A+K$$

$$\text{Let}\;E_{e}\left(\alpha ,1\right)=E_{e}\left(\alpha ,0\right)$$

$$\alpha =\frac{A+F}{F+3K}$$

Therefore, the Nash equilibrium between corporate shareholders and creditors is as follows: $\left(\alpha ,\beta \right)=\left(\frac{A+F}{F+3K},\frac{C}{2P}\right)$.

In the game matrix, shareholders might obtain financing by pledging their equity. While convenient, this method could transmit adverse signals, affecting stock prices (Berkman & Eleswarapu, 1998). On the other hand, creditors may choose to provide green bond investments to convey positive information, thereby enhancing the corporate social reputation (Bansal & Clelland, 2004; Flammer, 2013). However, they face the issues of uncertain returns and extended payback periods [11]; Ge & Liu, 2015).

RETRACTED

### 3.2 Game between shareholders and managers

Shareholders aim to maximize long-term corporate returns, while managers may prioritize immediate benefits, potentially avoiding projects requiring substantial resources, long payback periods, and high uncertainty. This discrepancy creates a principal-agent problem [6]. To incentivize managers, shareholders must evaluate their performance and implement compensation incentives. Under the EVA incentive system, rewards are based on actual EVA growth exceeding expectations [12]. Setting compensation based on EVA target benchmarks is necessary to avoid disputes. To measure green investments accurately, the calculation of GEVA is essential [36].

## 4 Case study

### 4.1 Background analysis of the case study

This study takes Nanjing Iron and Steel Co., Ltd. (NISCO, 600,282) as the case study. Established in 1999, NISCO's primary business involves the smelting and rolling of ferrous metals. As a heavy-polluting enterprise, it explicitly discloses its environmental expenditure, with environmental investments mainly used for low-carbon upgrades and renovations of equipment and sites. Furthermore, it provides a detailed disclosure of various data in the “Clean Production Evaluation System for the Steel Industry,” including comprehensive energy consumption per ton of steel, freshwater consumption per ton of steel, and sulfur dioxide emissions. These data serve as crucial foundations for calculating the enterprise's net profit after tax, debt capital, and equity capital, as well as the GEVA adjustment value calculated using the “Wolfe Weighting Method” (Wolfe & Linnenluecke, 2018). NISCO's comprehensive data and detailed environmental disclosure greatly benefit this research.

### 4.2 Calculation of the enterprise's economic value-added

#### 4.2.1 Net operating profit after tax (NOPAT) of NISCO

Table 2 shows the company's net operating profit after tax (NOPAT) of NISCO, which has seen a great rise since 2016 and has been stable.

#### 4.2.2 Total capital (TC)

The total capital of Nansteel Shareholding Enterprise includes equity capital and debt capital. When calculating, adjustments need to be made to the balance sheet items to reflect the actual invested capital, and the construction in progress should be excluded to prevent its long-term investment and short-term return characteristics from leading to negative EVA (Damodaran, 2007; Stern, Shiely & Ross, 2001).

We calculate and chart it according to the following formula.

The total capital is calculated as follows:

(4) TotalCapital=AverageOwners’Equity+AverageLiabilities−AverageInterest−freeCurrentLiabilities−AverageConstructioninProgress

The average interest-free current liabilities are calculated as follows:

(5) AverageInterest−freeCurrentLiabilities=AverageNotesPayable+AverageAccountsPayable+AverageEmployeeSalariesPayable+AverageTaxesPayable+AverageOtherPayables

The Total Capital (TC) is calculated as follows:

(6) TheTotalCapital(TC)=AverageShareholders’Equity+AverageLiabilities−AverageInterest−freeCurrentLiabilities−AverageConstructioninProgress

The statistical data are shown in Table 3.

RETRACTED

As can be seen from Table 3, the company's Average Interest-free Current Liabilities have been stable, while Average Salaries Payable and Average Taxes Payable have been on an upward trend.

Statistical data are shown in Tables 4 and 5

Table 4 shows that the company's Average Shareholders' Equity and Average Construction in Progress increased yearly while the Average Liabilities were stable.

Nanjing Iron & Steel's financing mainly comes from equity capital, especially equity pledges, with a relatively small proportion of debt capital. The impact of green investments on the reputation of equity pledges and the game will be discussed after considering environmental factors. Moreover, we calculate the pre-tax cost of debt capital of Nanjing Iron & Steel based on the one-year and five-year loan interest rates publicized by the People's Bank of China.

**Loans due within one year** are calculated as follows:

(7) Loansduewithinoneyear=Currentliabilities+Non−currentliabilitiesduewithinoneyear

Here, long-term loans include long-term loans and bonds payable, as shown in Table 6.

The GDP growth rate is shown in Table 7.

As calculated from the table：

The market risk premium for the year 2016： $R_{m}-R_{f}$ = 6.7%–1.5 % = 5.2 %

The market risk premium for the year 2017： $R_{m}-R_{f}$ = 6.9%–1.5 % = 5.4 %

The market risk premium for the year 2018: $R_{m}-R_{f}$ = 6.59%–1.5 % = 5.09 %

The market risk premium for the year 2019: $R_{m}-R_{f}$ = 6.1%–1.5 % = 4.6 %

The market risk premium for the year 2020: $R_{m}-R_{f}$ = 2.35%–1.5 % = 0.85 %

The market risk premium for the year 2021: $R_{m}-R_{f}$ = 8.1%–1.5 % = 6.6 %

The monthly β values for Nanjing Iron & Steel Co., Ltd. from 2016 to 2021 are shown in Table 8.

The cost of equity capital for Nanjing Iron and Steel Co., Ltd. from 2016 to 2021 is as shown in Table 9.

The cost of equity capital for Nanjing Iron and Steel Co., Ltd. is primarily derived through the Capital Asset Pricing Model (CAPM):

(8) $$R=R_{f}+\beta \left(R_{m}-R_{f}\right)$$

Through the above calculation of the cost and proportion of debt and equity capital for Nanjing Iron and Steel Co., Ltd., we have obtained the Weighted Average Cost of Capital (WACC). The weighted average cost of capital from 2016 to 2021 is shown in Table 10.

RETRACTED

#### 4.2.3 Economic Value Added

(9) AccordingtotheformulaEVA=NOPAT−TC*WACC

we calculate the Economic Value Added of Nanjing Iron and Steel Enterprise as shown in Table 11.

Nanjing Iron and Steel Enterprise emphasizes environmental investment in environmental protection, including capitalized expenditures that pay off long-term benefits at once, such as environmental protection equipment expenses and expenses that need to be amortized. However, the annual report does not disclose specific environmental expenditures. These data are provided by the Guotai'an Company's governance project, including the pollution discharge fees in the management expenses and the construction projects in progress in the notes to the financial statements, such as wastewater treatment and gas transformation projects.

As the subject of this study, Nanjing Iron & Steel Co., Ltd is a state-owned industrial enterprise under the central government, and its asset-liability ratio has been less than 75 % in recent years. Therefore, the capital cost rate in this study is calculated at 5.5 %. The asset-liability ratio of Nanjing Iron & Steel Co., Ltd from 2016 to 2020 is shown in Table 14.

### 4.3 Calculation of GEVA adjustment Value

#### 4.3.1 Calculation of environmental protection comprehensive score

The relevant environmental data of Nansteel Shares can be obtained from its annual report. Through the “Clean Production Evaluation Indicator System for the Steel Industry”, the standard values and actual values of Nansteel Shares were summarized and statistically displayed in the table, as shown in Table 15.

This study employs the “Wall gravity scoring method” to evaluate the environmental performance of Nansteel Share Co., Ltd., referring to the “Evaluation Index System of Clean Production in Steel Industry” to determine the standard and actual values of pollution indices. The Wall gravity scoring method is a method that combines the selected financial ratios with linear relationships, gives their respective score proportions, and then compares them with the standard ratios to determine the scores of each index and the cumulative scores of the overall index to evaluate the credit level of the enterprise. Wall gravity scoring is a method used to evaluate the relative importance of different factors. It evaluates the proportion of each indicator in the total score by assigning different weight values to more accurately reflect the characteristics of evaluation objects and results. This method is suitable for multi-dimensional and multi-index evaluation, can objectively and accurately reflect the evaluation object's advantages and disadvantages, and provides a scientific basis for decision-making. It further calculates the amount of environmental investment in the company's Economic Value Added (EVA) from 2016 to 2020. The evaluation process includes selecting indices and assigning weights, determining each index's standard and actual values, and calculating the results.

RETRACTED

The calculation formula is as follows:

(10) RelationshipRatio=1+(StandardValue−ActualValue)/StandardValue

Through comprehensive scoring and centralized evaluation, weights are assigned to different index elements at the weight allocation level, which are 25 %, 25 %, 25 %, 15 %, and 10 %, respectively, with a total weight of 100 %. The comprehensive scores of environmental effects from 2016 to 2020 are shown in Table 16.

Upon acquiring the comprehensive scores for Nansteel Shareholding Co., Ltd from 2016 to 2020 using the Vörösmarty Weighted Scoring Method, we can calculate the environmental cost rate by subtracting the standard 100 points from the total environmental protection score in the above table, then dividing by 100. Subsequently, by multiplying the environmental expense and capital expenditure by this environmental cost rate, we can ascertain the contributing expense cost and the contributing capital cost.

(11) TheadjustedvalueofGEVA=Contributingexpenseenvironmentalcost*(1−incometaxrate)+Contributingcapitalenvironmentalcost*costofcapitalratio

The calculation of the GEVA adjustment value from 2016 to 2020 is shown in Table 17.

#### 4.3.2 Calculation of GEVA

We have categorized and organized traditional EVA indicators and GEVA adjustment values based on the above computations. The sum of the GEVA adjustment value and the traditional EVA value determines the GEVA value. The values are shown in the following table, as shown in Table 18.

Nansteel's GEVA increased annually from 2016 to 2018, reaching 672,788.92 million yuan in 2018, reflecting the impact of government regulation and policy on enhancing GEVA. In 2016, the GEVA was negative, mainly due to low net profits, leading to negative post-tax net profit and traditional EVA. With the government's support for steel enterprises to resolve overcapacity and optimize business operations, Nansteel has increased its energy-saving and emission-reduction investments, promoting increased GEVA.

#### 4.3.3 Enterprise value evaluation model based on GEVA

The calculation of the green corporate value of Nansteel Shares from 2016 to 2020 is shown in Table 19.

The calculation formula for the green value of a company is:

(12) $$\sum_{t=1}^{\infty }\frac{NOPAT-\Delta TC+gEVA_{t}}{{\left(1+WACC\right)}^{t}}$$

According to the model established, we substitute the parameters into formula (12) for calculation.

$$2017：\frac{448812.5-\left(2290877.6-2115150.71\right)+31410.4}{1+6.9\%}=284841.92$$

$$2018：\frac{659822.4-\left(2674717.07-2290877.6\right)+12966.52}{1+6.87\%}=270374.71$$

$$2019：\frac{485205.64-\left(2888368.79-2674717.07\right)+82003.64}{1+6.49\%}=332010.1$$

$$2020：\frac{436078.68-\left(3229067.4-2888368.79\right)+58104.61}{1+2.55\%}=149668.14$$

RETRACTED

#### 4.3.4 Comparative advantage analysis of GEVA versus EVA

The above calculations compare the GEVA and the traditional EVA index, as shown in Table 20.

In 2016, both the EVA and GEVA of Nansteel Group were negative, indicating a lower investment in environmental protection. From 2017 to 2020, while environmental investments increased, the gap between EVA and GEVA remained small, suggesting that environmental efficiency was insignificant. Nonetheless, over the four years, Nansteel Group reduced pollutant indicators per ton of steel, such as sulfur dioxide emissions. GEVA was slightly higher than traditional EVA, reflecting its commitment to environmental protection while developing economically and enhancing its social responsibility. The GEVA was positive for all years, demonstrating that environmental investments did not lead to losses. Especially in 2019, environmental investments produced significant environmental benefits, further enhancing Nansteel Group's social responsibility and environmental protection advantages.

### 4.4 Analysis of the game between creditors' green debt investment and shareholders’ equity pledge financing

A comparison between the ecological value of the enterprise represented by GEVA and the adjusted value of GEVA is shown in Table 21.

From 2016 to 2020, the adjusted GEVA of Nansteel Group was consistently lower than the GEVA. Despite the small difference, it still reflected a positive value. After the steel industry was regulated in 2017, environmental issues received attention, but the effectiveness of Nansteel Group's green environmental investment was insignificant. In 2019, the adjusted GEVA reached 820,036.4 ten thousand yuan, which is notably high, displaying the potential for environmental investments to create positive value. The introduction of GEVA considered sustainable development and ecological benefits, not only focusing on economic benefits but also considering the opportunity cost of the ecological environment. The disclosure of corporate social responsibility reports demonstrates that corporations are placing more emphasis on social responsibility (Table 22).

This study investigates the game between shareholders' equity pledging and creditors' green investments. Equity pledging may damage the reputation and long-term development of the enterprise, while creditors tend to favor green investment to alleviate the negative impact of equity pledging. The adjusted value of GEVA considers the lag and uncertainty of green investment. It measures the performance of corporate environmental investment through the Walrasian weight scoring method and the calculation of environmental cost. The return obtained by shareholders through equity pledging is associated with the increase in the value of equity pledges within a year. Although equity pledging can quickly raise funds, its short-sightedness is not conducive to the enterprise's long-term development. Conversely, the enterprise's innovative investment, such as the capitalization of R&D investment, demonstrates its focus on long-term development, which can bring sustained returns.

(13) $$E_{g}=\left(\alpha ,\beta \right)=\alpha \left[\beta \left(-C+P\right)+\left(1-\beta \right)\left(-C\right)\right]+\left(1-\alpha \right)\left[\beta \left(-P\right)+\left(1-\beta \right)0\right]$$

The expected return of creditors in 2017 is as follows.

(1) The cost incurred by creditors investing in green bonds is C = 23601.07 ten thousand yuan.
(2) The profit P = 31410.4 ten thousand yuan for the company due to the good reputation brought by creditors' green investment.
(3) The return A = 28880.38 ten thousand yuan obtained by shareholders through equity pledging. (4) When shareholders pledge their equity not for short-term goals but for innovative long-term investment, the return from capitalization of R&D investment is F = 0.
(5) The loss K = −65436.71 ten thousand yuan was caused by the adverse development signals transmitted to the market by shareholders' equity pledging. The formula is as follows (equation (14)):

(14) α[β(23601.07+31410.4)+(1−β)(23601.01)+(1−α)[β(−31410.4)

According to equation (14), we let $E_{g}\left(1,\beta \right)=E_{g}\left(0,\beta \right)$ to obtain

$$\beta =\frac{C}{2P}=\frac{23601.07}{2*31310.4}=37.57\%$$

The expected shareholder return for 2017 is:

β[α(28880.38+65436.71)+(1−α)(28880.38−65436.71)+(1−β)[α(−65436.71)

$$\alpha =\frac{A+F}{F+3K}=14.71\%$$

The computation shows that the Nash equilibrium can be achieved when the game reaches its optimal state $\left(\alpha ,\beta \right)=\frac{A+F}{F+3K},\frac{C}{2P}$, ensuring the best possible outcome in the game.

RETRACTED

The expected investments of creditors in 2018 are as follows:

C (Cost of creditors investing in green bonds) = 15,022.21 ten thousand yuan.

P (Profits earned by the enterprise due to its good reputation from creditors’ green investment) = 12,966.52 ten thousand yuan.

A (Benefits obtained by shareholders through share pledging) = −152,616.82 ten thousand yuan F (Benefits brought by shareholders’ long-term innovative investment, i.e., capitalization of R&D input) = 0.

K (Losses caused by adverse market signals conveyed by shareholders’ share pledging) = 332,874.11 ten thousand yuan.

Similarly, the expected investment from shareholders in 2018 is as follows:

$\alpha =\frac{A+F}{F+3K}=\frac{-152616.82}{3*332874.11}=15.28\%$ The expected investment from creditors in 2019 is as follows:

(1) The cost incurred by the creditors for green bond investments, denoted as C, equals 35,563.84 ten-thousand yuan.
(2) The profits attributed to the company from the good reputation brought by green investments by creditors, denoted as P, equals 82,003.64 ten-thousand yuan.
(3) The profits obtained by shareholders through equity pledges, denoted as A, equals 98,987.42 ten thousand yuan.
(4) The profits brought by the dedication of shareholders to long-term innovation investments and capitalization of R&D expenses, denoted as F, equals 6849.9 ten thousand yuan.
(5) The loss caused by the unfavorable signals for development communicated to the market by shareholders' equity pledges, denoted as K, equals −253,857.02 ten-thousand yuan.

$\beta =\frac{C}{2P}=\frac{35563.84}{2*82003.64}=21.68\%\alpha =\frac{A+F}{F+3K}=\frac{98987.42+6849.9}{6849.9+3*\left(-253857.02\right)}=14.02\%$ Therefore, the expected investment by shareholders in 2019 is as follows:

The expected investment by creditors in 2020 is as follows:

C (cost incurred by creditors investing in green bonds) = 43,164.16 ten thousand yuan.

P (profits obtained by the company due to the positive reputation from creditors’ green investment) = 58,104.61 ten thousand yuan.

A (returns obtained by shareholders from pledging equity) = −93,305.06 ten thousand yuan.

F (returns from innovative long-term investment, i.e., capitalization of R&D input) = 5139.48 ten thousand yuan.

K (loss caused by the negative signal to the market due to shareholders’ equity pledge) = 196,697.16 ten thousand yuan.

The expected investment by shareholders in 2020: $\beta =\frac{C}{2P}=\frac{43164.16}{2*58104.61}=37.14\%$.

The research indicates that the probability of equity pledging financing by Nansteel Group exceeds that of green investments by creditors. Although eco-investments enhance corporate social responsibility image, equity financing is still more popular. An increase in equity pledging will lead to a rise in the cost of green debt, while its reduction will decrease the cost. Even though green bond investment can mitigate the impact of equity pledging on corporate reputation, its effectiveness is insignificant. Nansteel Group still has room for improvement in awareness and motivation toward green investments.

RETRACTED

Additionally, the quantity of equity pledging does not significantly drive corporate innovation. While green bond investment can alleviate the impact of equity pledging on reputation, its effectiveness is not pronounced. The study also employs game theory models and EVA return rate to evaluate corporate performance, eliminating the impact of capital size on the results.

β represents the probability of corporate shareholders investing in eco-projects,

TC stands for the total capital of the enterprise.

(15) $$\text{Green}\;\text{EVA}\;\text{Return}\;\text{Rate}=\frac{GreenEVA}{TC}\times \beta =\frac{EVA+\text{Green}\;\text{EVA}\;\text{Adjustment}\;\text{Value}}{TC}\times \beta$$

(16) $$\text{EVA}\;\text{Return}\;\text{Rate}=\frac{EVA}{TC}\left(1-\beta \right)$$

We respectively calculated the corporate GEVA rate of return and EVA rate of return from 2016 to 2020, as shown in Table 23.

When the GEVA Return Rate > EVA Return Rate.

2016：-1.31β＞-1.47（1-β） β＞0.53。

2017：20.96β＞19.59（1-β） β＞48.31 %。

2018：25.15β＞24.67（1-β） β＞0.5。

2019：19.64β＞16.8（1-β） β＞0.46。

2020：15.3β＞13.5（1-β） β＞0.47。

The probability of green environmental investment in Nansteel was substantial in 2016 but dropped below 50 % in 2017, 2019, and 2020. This was primarily due to a defensive search for new transformations, such as environmental investments, in the context of a negative traditional EVA. However, in a profitable state, management protects current interests and avoids long-term and lagging investments. The gap between GEVA and traditional EVA is determined by environmental expenditure, with Nansteel's capitalization of environmental expenditures being higher than their expense-based spending. However, overall, the company's desire for environmental investments is not high, and creditors focus more on current benefits, placing little emphasis on the return from environmental investments.

### 4.5 The impact of GEVA development on carbon emissions

The development of GEVA has a positive impact on reducing carbon emissions. Firstly, it innovates the corporate environmental governance model, providing guarantees for green development and promoting government attention to low-carbon environmental issues. Secondly, businesses focusing on GEVA can stimulate the development of the tertiary sector, triggering a shift in consumer attitudes and placing more emphasis on whether a product is environmentally friendly. This enhances public environmental awareness and the concept of green consumption, further reducing corporate carbon emissions. In the 21st century, the concept of green and sustainable economic development has been widely disseminated. Green transformation guides resource conservation and environmentally friendly development, with green innovation at the core, considering both environmental and economic benefits. The development of GEVA will lower carbon emission intensity and effectively promote the transition to a low-carbon economy and green economic development.

RETRACTED

## 5 Conclusions and outlook

### 5.1 Conclusion and suggestion

#### 5.1.1 Conclusion

Green investment plays a significant role in promoting environmental protection, and it represents an active and forward-looking investment strategy that emphasizes the protection and improvement of the ecological environment. However, since green investment usually requires a large amount of capital investment and the payback period is relatively long, the uncertainty of its investment return challenges enterprises' reputation management. Green performance and creditor investment can undoubtedly enhance the company's public image, making the company more attractive in the eyes of investors, thus stimulating the stock price. However, at the same time, we must also face up to the problem. When shareholders are under financial pressure, they may pledge their shares to secure financing, a practice that can raise various financial and agency issues.

Although equity pledge financing can provide financial support quickly, this financing method may interfere with enterprises' normal decision-making process and may even make enterprises pay too much attention to short-term interests while ignoring long-term development. In order to mitigate this impact, this study uses a game theory model to analyze creditors’ green bond investment decisions to find a way to mitigate the impact of equity pledge financing on corporate reputation. The results of the analysis show that although green investment can help enterprises improve their reputation, enterprises are more inclined to choose equity pledge financing because of the convenience of equity pledge financing. However, this does not mean we should ignore the importance of green investment. In fact, with the increasing emphasis on environmental protection, green performance and investment have become an important part of corporate reputation.

As a performance evaluation indicator, GEVA pays attention to the economic benefits of enterprises, social benefits, and environmental protection. By introducing GEVA, we can optimize business management, improve efficiency, protect the environment, and maximize benefits. However, principal-agent problems may arise due to the differences in the interests of capital providers and the differences in the development goals of enterprises. In addition, due to the delayed nature of GEVA and the long payback period of green investment, it is not easy to accurately evaluate its environmental benefits in the short term, which may encourage enterprises to pursue immediate benefits and ignore environmental protection. Therefore, how to solve this problem so that enterprises pursue economic benefits at the same time but also fulfill environmental responsibility actively is the direction we need in-depth research.

RETRACTED

As an objective measure of the company's operating conditions, EVA rate of return can reflect the profitability of a company and the degree of protection of shareholders' interests. However, excessive focus on EVA returns may cause companies to ignore the value of ecological resources and even harm the interests of shareholders. Taking Nangang as an example, its GEVA return rate is higher than the EVA return rate, which indicates that Nangang's investment in environmental protection has brought considerable economic return. This is further evidence that environmental investments can create value rather than necessarily increasing EVA returns at the expense of the environment. It also reminds us that the success of an enterprise lies not only in short-term economic gains but also in long-term sustainable development and social responsibility fulfillment.

The added value of a green economy is a kind of index that can reflect the enterprise's environmental input and environmental protection contribution. By introducing GEVA, we can better measure companies' environmental efforts and investments while encouraging companies to pay more attention to environmental protection and social responsibility. However, in practice, major shareholders are often more inclined to obtain financing through equity pledges to meet their capital needs rather than choose to make green investments. This phenomenon may be related to creditors' investment preferences, policy incentives, and market environment. Future studies should further explore how to encourage all parties to actively participate in green investment through policy guidance, market mechanisms, and other means, and how to balance the interests of all capital providers through green economic added value (GEVA) to encourage more parties to participate in green investment and promote enterprises to pay more attention to environmental protection and social responsibility.

#### 5.1.2 Suggestions

Explore diversified financing methods: Since equity pledge financing has negative effects, such as interfering with corporate decision-making and causing financial and agency problems, enterprises should actively explore diversified financing methods. For example, we can try to issue green bonds and carry out green project cooperation for financing to reduce the impact of equity pledge financing on corporate reputation.

RETRACTED

Strengthen policy incentives: Governments can introduce policies encouraging companies to invest in green. For example, tax incentives and subsidies will be given to enterprises that carry out green investment, while supervision and law enforcement on environmental protection will be strengthened to ensure that enterprises truly achieve the goal of green investment.

Establish green investment standards: Green investment standards or guidelines can be established to make green investment more regulated and transparent. These standards or guidelines can clarify the scope, evaluation indicators, and methods of green investment to help enterprises and investors better understand and practice green investment.

Improve the environmental awareness of enterprises: enterprises should strengthen the cultivation of environmental awareness and improve the importance of environmental protection. At the same time, enterprise leaders should fully recognize the importance and long-term benefits of green investment and actively promote enterprises’ green transformation and sustainable development.

Strengthen investor education: Investors should pay more attention to companies' environmental behavior and green investment plans and strengthen the evaluation and investigation of these aspects. At the same time, the government and regulators should also strengthen investors’ education to help them better understand the risks and benefits of green investment to promote the healthy development of green investment.

Research on green investment strategies: Given that major shareholders are more inclined to equity pledge financing, we can further study the strategies and methods of green investment. For example, how to achieve the sustainable development goals of enterprises through green project investment, environmental technology innovation, and other ways while improving the market value and competitiveness of enterprises.

Play the role of industry associations: Industry associations can play their organizational and guiding roles to promote green cooperation and exchanges among enterprises. For example, activities such as green investment forums and environmental technology exchanges can be organized to provide enterprises with more green investment opportunities and partners.

In short, in order to promote the green investment and sustainable development of enterprises, it is necessary for the government, enterprises, investors, and all sectors of society to work together to form a diversified and all-round promotion mechanism.

RETRACTED

### 5.2 Research limitations

Green EVA considers environmental input, reflecting corporate performance, but it has limitations as it is easily influenced by human manipulation, which may be detrimental to corporate development. Using Nansteel as an example, this study showcases the game among capital providers and finds that corporate financing tends to lean toward shareholders' equity pledging financing. Although creditors have green investments to mitigate the negative effects of equity pledging, their impact is small. Therefore, it is necessary to incentivize corporate green bond investments positively, improve their social status and reputation, and encourage green investment. However, the difficulty of obtaining environmental data and information on corporate environmental expenditure, as well as insufficient voluntary disclosure, also affects the accuracy of GEVA. Moreover, major shareholders’ equity pledging might lead enterprises to focus excessively on short-term gains, overlooking long-term development and innovation. Hence, it is necessary to design a more reasonable GEVA performance mechanism and stimulate capital providers to pay attention to environmental benefits while pursuing economic benefits through wage and salary incentives.

### 5.3 Outlook and future

This study deeply explores the comprehensive evaluation of the game among corporate capital providers from the perspective of GEVA. GEVA emphasizes the importance of environmental protection and social responsibility while pursuing profits, achieving both economic and environmental win-win. The article reveals that while capital providers pay attention to corporate profits, they are more concerned about fulfilling environmental protection and social responsibility. As a comprehensive evaluation indicator that includes corporate economic, environmental, and social benefits, GEVA helps enterprises fully evaluate their performance. GEVA is expected to be widely applied in corporate performance evaluation and investment decision-making, promoting the sustainable development of the economy, environment, and society. It has certain reference significance for the financing methods of heavily polluting enterprises.

## Data availability statement

The data supporting this study's findings are available from the corresponding author upon reasonable request.

## Funding information

The author(s) disclosed receipt of the following financial support for the research, authorship, and/or publication of this manuscript:

10.13039/100018978Zhejiang Office of Philosophy and Social Science, China (Grant/Award Number: 23NDJC154YB).

RETRACTED

Study on the Course Module Design and Teaching Model Reform for Training Excellent Accounting Talents under the Convergence of ‘Dual Carbon’ Goals and ‘Digital Economy’—a Graduate Teaching Reform Project of the Zhejiang Province's 14th Five-Year Plan.

10.13039/100022963General Research Project of Zhejiang Provincial Department of Education, China (No. 2023-005) and the 10.13039/501100008867Zhejiang Graduate Education Society, China (No. 2023-005).

## CRediT authorship contribution statement

**Wunhong Su:** Writing – review & editing, Supervision, Conceptualization. **Quansheng Zhang:** Writing – original draft. **Yunxia Ling:** Methodology. **Wong Ming Wong:** Investigation, Formal analysis.

## Declaration of competing interest

All authors declare that No conflict of interest exists.

## Figures and Tables

**Table 1:** Creditor and Shareholder Game Matrix

	Shareholder Increases Equity Pledge (Shareholder) β	Shareholder Does Not Increase Equity Pledge (Shareholder)（1-β）
Creditor Increases Green Bond Investment (Creditor) α	-C + P,A-K	-C, F + K
Creditor Does Not Increase Green Bond Investment (1-α)	-P, A + K	0,0

Table by authors.

**Table 2:** Calculation Table of Net Profit After Tax Unit: 10,000 Yuan

Item/Year	2016	2017	2018	2019	2020	2021
Net Profit	35488.5	340068.77	474089.09	336485.52	318755.28	409518.48
Minority Shareholder's Income	114.98	20033.83	73269.22	75863.08	34163.78	418.18
Capitalized R&D Investment	0	0	0	6849.9	5139.48	14370.56
Interest Expense	74093.08	60612.15	42138.65	36260.34	43774.25	41243.14
Impairment Loss on Various Assets	14352.55	36904.44	31069.74	32775.97	23237.5	38601.32
Non-operating Expenditure	1556.48	13099.5	13478.83	17023.08	2623.76	9303.39
Non-operating Income	15772.91	835.6	658.92	1615.91	4434.67	4351.23
Increase in Deferred Income Tax Liabilities	3669.61	0	1582.66	3313.8	7032.93	5455.29
Increase in Deferred Income Tax Assets	−8079.93	−6374.54	−46360.2	639.27	−22086.58	−2676.17
Net Operating Profit After Taxes (NOPAT)	103024.92	448812.5	659822.4	485205.64	436078.68	496036.15

As shown in Table 2, the Net Operating Profit After Taxes (NOPAT) is calculated as follows: NOPAT = Net Profit + Minority Shareholder's Income + Capitalized R&D Investment + (Interest Expense + Impairment Loss on Various Assets + Non-operating Expenditure - Non-operating Income) * (1 - Income Tax Rate) + Increase in Deferred Income Tax Liabilities - Increase in Deferred Income Tax Assets (Damodaran, 2007). Table by authors.

**Table 3:** Calculation Table of Average Interest-free Current Liabilities Unit: 10,000 Yuan

Item/Year	2016	2017	2018	2019	2020	2021
Average Notes Payable	713641.22	681828.89	609571.95	613476.56	558348.28	665715.75
Average Accounts Payable	432329.45	433706.32	405558.81	393972.95	403952.82	445136.1
Average Salaries Payable	25106.95	47432.3	69903.91	74675.86	75156.36	73414.15
Average Taxes Payable	11417.79	18615.32	54144.42	60669.45	38402.61	43035.07
Average Other Payables	179631.35	73790.76	36435.2	31500.94	33527.16	45888.35
Average Interest-free Current Liabilities	1362126.76	1255373.59	1175614.29	1174295.76	1109387.23	1273189.42

Table by authors The Total Capital (TC) = Average Shareholders' Equity + Average Liabilities - Average Interest-free Current Liabilities - Average Construction in Progress (6).

RETRACTED

**Table 4:** Calculation Table for Total Capital Unit: 10,000 RMB

Items/Years	2016	2017	2018	2019	2020	2021
Average Shareholders' Equity	655790.29	1117693.42	1768390.75	2087051.7	2303941.1	1619050.17
Average Liabilities	2876463.17	2484161.08	2178110.77	2153703.3	2272398.9	2382524.51
Average Construction in Progress	54975.99	55603.27	96170.16	178090.45	237885.37	240071.7
Average Interest-Free Current Liabilities	1362126.76	1255373.59	1175614.29	1174295.76	1109387.2	1273189.42
Total Capital	2115150.71	2290877.6	2674717.07	2888368.79	3229067.4	2488313.56

Table by authors.

**Table 5:** Total Capital Calculation Unit: Ten thousand yuan

Items/Years	2016	2017	2018	2019	2020	2021
Short-term Loans	776625.91	330398.81	489725.52	343605.73	449899.1	449899.1
Long-term Loans	4400	71876.2	7600	84520.08	124611.59	124611.59
Non-current Liabilities Due Within One Year	94045.85	286239.03	86,190	10,100	18,250	21074.99
Bonds Payable	277831.41	398633.33	277831.41	102652.2	154006.73	51322.43
Debt Capital	1152903.17	1087147.37	861346.93	540878.01	746767.42	646908.11
Equity Capital	2277261.38	2686397.06	3258111.67	3821173.34	4043861.17	5123187.39
Total Capital	3430164.55	3773544.43	4119458.6	4362051.35	4790628.59	5770095.5
Debt Capital Ratio	33.61 %	28.8 %	20.9 %	12.4 %	15.6 %	11.21 %
Equity Capital Ratio	66.39 %	71.2 %	79.1 %	87.6 %	84.4 %	88.79 %

Table by authors.

**Table 6:** Calculation Table for After-tax Cost of Debt Capital

Item/Year	2016	2017	2018	2019	2020	2021
Weight of Loans Due within One Year in Debt Capital	75.52 %	56.72 %	66.86 %	65.39 %	62.69 %	80.74 %
Weight of Long-term Loans in Debt Capital	24.48 %	32.16 %	7.46 %	34.6 %	37.3 %	19.26 %
One-Year Bank Loan Interest Rate	4.35 %	4.35 %	4.35 %	4.35 %	4.35 %	4.35 %
Five-Year Bank Loan Interest Rate	4.75 %	4.75 %	4.75 %	4.75 %	4.75 %	4.75 %
Pre-tax Cost of Debt Capital	4.45 %	3.99 %	3.26 %	4.49 %	4.5 %	4.43 %
After-tax Cost of Debt Capital	3.34 %	3 %	2.45 %	3.37 %	3.37 %	3.32 %

Table by authors Loans due within one year = Current liabilities + Non-current liabilities due within one year(7).

RETRACTED

**Table 7:** GDP Growth Rate from 2016 to 2021

	2016	2017	2018	2019	2020	2021
GDP Growth Rate	6.7 %	6.9 %	6.59 %	6.1 %	2.35 %	8.1 %

Table by authors.

**Table 8:** Monthly β Values for Nanjing Iron & Steel Co., Ltd., 2016–2021

	2016	2017	2018	2019	2020	2021
January	1.24157	1.26144	1.30422	1.35768	1.08421	1.01063
February	1.24115	1.26375	1.26434	1.34014	1.08808	1.01372
March	1.21673	1.266	1.29548	1.19942	1.11503	0.97124
April	1.21529	1.26641	1.2762	1.2106	1.10199	0.96115
May	1.22079	1.28475	1.27901	1.24522	1.09437	0.87806
June	1.21367	1.28466	1.24769	1.28501	1.17819	0.84481
July	1.20549	1.3097	1.26651	1.13139	1.01352	0.67905
August	1.21195	1.31873	1.29039	1.14381	0.98424	0.68672
September	1.2122	1.32758	1.26713	1.11325	0.98344	0.67546
October	1.21557	1.32557	1.2658	1.04506	0.99074	0.70647
November	1.22832	1.30191	1.297	1.04906	0.98308	0.75747
December	1.24768	1.31423	1.35663	1.05051	1.03298	0.7569
Average	1.2225	1.2937	1.2842	1.1809	1.0542	0.82847

Table by authors.

**Table 9:** Cost of Equity Capital for Nanjing Iron and Steel Co., Ltd. from 2016 to 2021

Items/Year	2016	2017	2018	2019	2020	2021
Risk-free Rate of Return ($R_{f}$)	1.5 %	1.5 %	1.5 %	1.5 %	1.5 %	1.5 %
Market Risk Premium ($R_{m}-R_{f}$)	5.2 %	5.4 %	5.09 %	4.6 %	0.85 %	6.6 %
β Value	1.2225	1.2937	1.2842	1.1809	1.0542	0.8285
Cost of Equity Capital	7.86 %	8.49 %	8.04 %	6.93 %	2.4 %	6.97 %

Table by authors.

**Table 10:** Weighted Average Cost of Capital (WACC), 2016–2021

Item/Year	2016	2017	2018	2019	2020	2021
Debt Capital Ratio	33.61 %	28.8 %	20.9 %	12.4 %	15.6 %	11.21 %
Cost of Debt Capital	3.34 %	3 %	2.45 %	3.37 %	3.37 %	3.32 %
Equity Capital Ratio	66.39 %	71.2 %	79.1 %	87.6 %	84.4 %	88.79 %
Cost of Equity Capital	7.86 %	8.49 %	8.04 %	6.93 %	2.4 %	6.97 %
Weighted Average Cost of Capital	6.34 %	6.9 %	6.87 %	6.49 %	2.55 %	6.56 %

Table by authors $R=R_{f}+\beta \left(R_{m}-R_{f}\right)$ (8).

**Table 11:** Calculation of Economic Value Added Unit: 10,000 yuan

Item/Year	2016	2017	2018	2019	2020	2021
NOPAT	103024.92	448812.5	659822.4	485205.64	436078.68	496036.15
TC	2115150.71	2290877.6	2674717.07	2888368.79	3229067.4	2488313.56
WACC	6.34 %	6.9 %	6.87 %	6.49 %	2.55 %	6.56 %
EVA	−31075.64	290741.95	476069.34	297750.51	353737.46	332802.78

Table by authors EVA = NOPAT - TC*WACC (9).

**Table 12:** Calculation Table of Environmental Input Costs from 2016 to 2020 Unit: 10,000 yuan

Item/Year	2016	2017	2018	2019	2020
Expensed Costs	7925.61	71,437	23,926	167,611	117,443
Capitalized Costs	10904.7	10511.16	47950.6	119194.2	159250.32
Environmental Costs	18830.31	81948.16	71876.6	286805.2	276693.32

Table by authors.

**Table 13:** Total Environmental Costs and Net Profit of Nansteel Co., Ltd. from 2016 to 2020

Items/Years	2016	2017	2018	2019	2020
Net Profit	35488.5	340068.77	474089.09	336485.52	318755.28
Environmental Costs	18830.31	81948.16	71876.6	286805.2	276693.32

Table by authors.

RETRACTED

**Table 14:** Asset-Liability Ratio of Nanjing Iron & Steel Co., Ltd from 2016 to 2020

Item/Year	2016	2017	2018	2019	2020
Asset-Liability Ratio	80.19 %	58.77 %	51.91 %	49.72 %	49.59 %
Cost of Equity Capital Rate	5.5 %	5.5 %	5.5 %	5.5 %	5.5 %

Table by authors.

**Table 15:** Actual and Standard Values of Ton Steel Energy Consumption for Each Project

Items	Units	Standard Value	2016 Actual Value	2017 Actual Value	2018 Actual Value	2019 Actual Value	2020 Actual Value
Comprehensive Energy Consumption per Ton of Steel	Kgce/t steel	≤680	589.8	572	555.3	553.7	551.7
Fresh Water Consumption per Ton of Steel	$m^{3}/t$ steel %	≤6	3.1	2.6	1.95	1.82	1.98
Sulfur Dioxide Emission per Ton of Steel	Kg/t steel	≤1	0.43	0.3	0.28	0.28	0.13
Smoke Dust Emission per Ton of Steel	Kg/t steel	≤3	0.53	0.45	0.16	0.64	0.79
COD Emission per Ton of Steel	Kg/t steel	≤0.2	0.018	0.016	0.007	0.007	0.009

Table by authors.

**Table 16:** Calculation of Comprehensive Scores for Environmental Effects from 2016 to 2020

Items	Comprehensive Energy Consumption per Ton of Steel	Fresh Water Consumption per Ton of Steel	Sulfur Dioxide Emissions per Ton of Steel	Dust Emissions per Ton of Steel	COD Emissions per Ton of Steel	Comprehensive Score
Weight	25	25	25	15	10	100
2016 Relationship Ratio	1.12	1.48	1.57	1.82	1.91	–
2016 Relationship Score	28	37	39.25	27.3	19.1	150.65
2017 Relationship Ratio	1.16	1.57	1.7	1.85	1.92	–
2017 Relationship Score	29	39.25	42.5	27.75	19.2	157.7
2018 Relationship Ratio	1.18	1.68	1.72	1.95	1.97	–
2018 Relationship Score	29.5	42	43	29.25	19.7	163.45
2019 Relationship Ratio	1.19	1.7	1.72	1.79	1.97	–
2019 Relationship Score	29.75	42.5	43	26.85	19.7	161.8
2020 Relationship Ratio	1.19	1.67	1.7	1.74	1.97	–
2020 Relationship Score	29.75	41.75	42.5	26.1	19.7	159.8

Table by authors Relationship Ratio = 1+(Standard Value-Actual Value)/Standard Value (10).

**Table 17:** Calculation of GEVA Adjustment Value for Nansteel Shareholding Co., Ltd from 2016 to 2020

Item	2016	2017	2018	2019	2020
Expense Cost (10,000 CNY)	7925.61	71,437	23,926	167,611	117,443
Capital Cost (10,000 CNY)	10904.7	10511.16	47950.6	119194.2	159250.32
Comprehensive Score	150.65	157.7	163.45	161.8	159.8
Environmental Cost Rate	0.5	0.58	0.63	0.62	0.6
Contributing Expense Environmental Cost (10,000 CNY)	3962.81	41433.46	15073.38	103918.82	70465.8
Contributing Capital Environmental Cost (10,000 CNY)	5452.35	6096.47	30208.88	73900.4	95550.19
Income Tax Rate	25 %	25 %	25 %	25 %	25 %
Cost of Capital Rate	5.5 %	5.5 %	5.5 %	5.5 %	5.5 %
GEVA Adjustment Value	3271.99	31410.4	12966.52	82003.64	58104.61

Table by authors The adjusted value of GEVA = Contributing expense environmental cost * (1- income tax rate) + Contributing capital environmental cost * cost of capital ratio (11).

RETRACTED

**Table 18:** Calculation of GEVA for Nansteel Shares, 2016–2020 Units: 10,000 CNY

Item/Year	2016	2017	2018	2019	2020
EVA	−31075.64	448812.5	659822.4	485205.64	436078.68
GEVA Adjustment Value	3271.99	31410.4	12966.52	82003.64	58104.61
GEVA	−27803.65	480222.9	672788.92	567209.28	494183.29

Table by authors.

**Table 19:** Calculation of the Green Corporate Value of Nansteel Shares, 2016–2020 Units: 10,000 CNY

Item/Year	2016	2017	2018	2019	2020
NOPAT	103024.92	448812.5	659822.4	485205.64	436078.68
TC	2115150.71	2290877.6	2674717.07	2888368.79	3229067.4
WACC	6.34 %	6.9 %	6.87 %	6.49 %	2.55 %
EVA	−31075.64	290741.95	476069.34	297750.51	353737.46
GEVA Adjustment Value	3271.99	31410.4	12966.52	82003.64	58104.61
GEVA	−27803.65	480222.9	672788.92	567209.28	494183.29

Table by authors.

Table by authors $\sum_{t=1}^{\infty }\frac{NOPAT-\Delta TC+gEVA_{t}}{{\left(1+WACC\right)}^{t}}$ (12).

**Table 20:** Comparison of EVA and GEVA Values from 2016 to 2020 Units: 10,000 yuan

	2016	2017	2018	2019	2020
EVA (Ten thousand yuan)	−31075.64	448812.5	659822.4	485205.64	436078.68
GEVA (Ten thousand yuan)	−27803.65	480222.9	672788.92	567209.28	494183.29

Table by authors.

**Table 21:** Comparison of EVA Adjusted Values and GEVA Values from 2016 to 2020 Unit: Ten thousand yuan

	2016	2017	2018	2019	2020
GEVA Adjustment Value	3271.99	31410.4	12966.52	82003.64	58104.61
GEVA	−27803.65	480222.9	672788.92	567209.28	494183.29

Table by authors.

**Table 22:** Evaluation of the Game between Green Debt Investment and Equity Pledge from 2017 to 2020 Unit: Ten thousand yuan

Item/Year	2017	2018	2019	2020
The proportion of Debt Capital	28.8 %	20.9 %	12.4 %	15.6 %
Environmental Cost	81948.16	71876.6	286805.2	276693.32
Green Debt Cost for Creditors	23601.07	15022.21	35563.84	43164.16
Increase in GEVA from the Previous Year	508026.55	192566.02	−105579.64	−73025.99
Increase in Debt Capital GEVA from the Previous Year	146311.65	40246.3	−13091.88	−11392.05
Increase in Equity Pledges from the Previous Year	367,621,958	−1681,172,286	1,681,172,286	−1681,172,286
Earnings per Share	0.7856	0.9078	0.5888	0.555
Return from Equity Pledges	28880.38	−152616.82	98987.42	−93305.06
Adjusted Value of GEVA	31410.4	12966.52	82003.64	58104.61
Capitalization of R&D Investment	0	0	6849.9	5139.48
Social Contribution per Share	1.78	1.98	1.51	1.17
Loss Caused by Adverse Signals from Equity Pledge	−65436.71	332874.11	−253857.02	196697.16

Table by authors.

RETRACTED

**Table 23:** Calculation Table for GEVA Return Rate and EVA Return Rate, 2016–2020 Unit: Ten thousand yuan

Items	2016	2018	2019	2020
Total Capital (TC)	2115150.71	2674717.07	2888368.79	3229067.4
EVA	−31075.64	659822.4	485205.64	436078.68
GEVA	−27803.65	672788.92	567209.28	494183.29
EVA Return Rate	−1.47 %	24.67 %	16.8 %	13.5 %
GEVA Return Rate	−1.31 %	25.15 %	19.64 %	15.3 %

Table by authors.

$\text{Green}\;\text{EVA}\;\text{Return}\;\text{Rate}=\frac{GreenEVA}{TC}\times \beta =\frac{EVA+\text{Green}\;\text{EVA}\;\text{Adjustment}\;\text{Value}}{TC}\times \beta$ (15).

$\text{EVA}\;\text{Return}\;\text{Rate}=\frac{EVA}{TC}\left(1-\beta \right)$ (16).
